The article "Function Mechanism of Psychological Driving Factors and Professional Transformation: Migrant Workers to Industrial Workers" was published in 2022. Journal: J Environ Public Health.

# Function Mechanism of Psychological Driving Factors and Professional Transformation: Migrant Workers to Industrial Workers

**DOI:** 10.1155/2022/9686998

**Published:** 2022-08-31

**Authors:** Su Yang, Tianyue Tang, Hongyang Li, Long Zhu, Jiawei Huang

**Affiliations:** ^1^School of Economics and Management, Anhui Jianzhu University, Hefei 230022, China; ^2^Anhui Province Center for Migrant Workers Studies, Fuyang Normal University, Fuyang 236000, China; ^3^Anhui Province Construction Economy and Real Estate Management Research Center, Hefei 230022, China; ^4^Business School of HOHAI University, Nanjing 211100, China

## Abstract

With in-depth development of industrialization and urbanization in China, improving the professional skills and quality of migrant workers in the construction industry has become an important measure to optimize the labor force structure and promote the industry upgrading. Numerous studies have been carried out on this topic, and construction industrial workers with high skills level and professional quality have replaced the professional identity of migrant workers. However, the psychological cognitive mechanism of migrant workers' occupational role enhancement behavior has not been fully revealed. This study aims to construct a theoretical model of the intention to influence the industrialization of migrant workers in the construction industry based on the frameworks of the theory of planned behavior and risk perception theory, and to explore the key factors and cognitive mechanisms in their transformation into industrial workers in the construction industry. Empirical study using structural equation modeling through field collection of 383 questionnaires from migrant construction workers shows that perceived behavioral control, subjective norm, and behavioral attitude all have significant positive effects on behavioral intention, with decreasing direct effects in descending order of magnitude. Perceived behavioral control also predicts professionalization through the mediation of behavioral intentions, and the newly introduced risk perception factor in the model has a negative inhibitory effect on behavioral intentions and actual behavior. This study validates the important role of psychological intention on the industrialization of migrant workers in the construction industry, providing a new perspective to promote their transformation into industrial workers, and laying the foundation for the modern transformation and sustainable industry development.

## 1. Introduction

In modern society, occupation is a fundamental dimension of social stratification and affects personal development and social stability. In the rapid industrialization and urbanization, migrant workers, as a unique product of China's dualistic economic system [1], have a rural household registration and are engaged in nonagricultural industries in the city. By doing so, they earn labor income and social value. The ambiguous status of “half-farmers and half-workers” has resulted in this group not being able to enjoy the education and medical resources of urban residents. This status has created an awkward position for migrant workers [2], and the solution to their problems still requires a return to their socially productive status [3]. According to Marx's theory of class analysis, the state of possession of a social subject in the means of social production determines its class attributes. Raising the value of its own occupational identity and increasing that of migrant workers are the fundamental way to solve the contradictions of migrant workers.

The article "Function Mechanism of Psychological Driving Factors and Professional Transformation: Migrant Workers to Industrial Workers" was published in 2022. Journal: J Environ Public Health.

As a pillar industry of China's economy, the construction industry absorbs nearly 50 million migrant workers every year, which is second only to the manufacturing industry. In recent years, the construction industry is undergoing a critical stage of transformation and development, with advanced production equipment, construction concepts, and technologies gradually applied in production practices. However, the professionalism of the workforce cannot match its transformation and development needs; thus, problems arise such as low workforce quality, severe ageing, and serious loss of highly skilled workers [4, 5]. In addition, construction work is labor-intensive, high risk, and has poor environmental conditions and high pressures that lead to difficulties in attracting young workers. Low-quality labor resources are no longer sufficient to meet the transformational development of the construction industry and cause an urgent need for a group of construction industry workers with high technical quality, stable positions, high social status, and legal labor security rights.

The professional transformation of jobs has been considered to be the most beneficial to improve the overall professional quality of workers and promote the industry upgrading and development. William E. Snizek pointed out that with the continuous societal development, more industries join the professional transformation, which becomes an important sign to judge their maturity [6]. At present, research on the transformation of industrial workers in the construction industry mainly focuses on the influencing factors. Considering the industry participants as the research perspective from the macro level, this study finds that macro policies, enterprise management, and human capital investment all have a significant effect on the cultivation of industrial workers in the construction industry. However, research on the motivation behind individual professional transformation is relatively weak. As the main subject of professional transformation, the behavioral changes of migrant workers in the frontline construction industry directly affect its transformation and development. Then, what are the key factors that influence the behavior of migrant workers' industrialization? What needs to be done to motivate migrant workers in the construction industry to become industrial workers? Only by sorting out the cognitive, attitudinal, self-awareness, and other psychological factors behind the behavior, combined with the external context, can the driving mechanism of the industrialization of migrant workers in the construction industry be systematically examined. Therefore, this study refers to the theory of planned behavior and of risk perception to construct a research framework that provides a new perspective and empirical support to better understand the psychological mechanism of the professional transformation of migrant workers in the construction industry.

The article "Function Mechanism of Psychological Driving Factors and Professional Transformation: Migrant Workers to Industrial Workers" was published in 2022. Journal: J Environ Public Health.

## 2. Literature Review

Theory of planned behavior (TPB) was developed by Ajzen in 1991 as an important predictive model for the study of individual behavior in social psychology [7], based on theory of reasoned action (TRA) [8], with the addition of perceptual behavioral control (PBC). The theoretical model is illustrated in Figure 1. Attitude (AT) is an individual's positive or negative evaluation of a particular behavior. Subjective norm (SN) is the perceived pressure of significant others or groups to perform a particular behavior. Perceived behavioral control (PBC) is an individual's perception of the ability to control the resources and opportunities needed to perform a particular behavior. TPB considers behavioral intention (BI) as a direct psychological factor influencing behavior, which can be affected by AT, SN, and PBC. In addition, PBC can also have a nonvolitional influence on behavior, which compensates for the fact that TRA only considers volitional influences. Therefore, according to TPB, the more positive an individual's AT toward the behavior, the more that SN supports engaging in the behavior, while the stronger PBC over the behavior, the higher the individual's BI. TPB explains individual intention to influence behavioral processes from the perspective of information processing and expectancy theory, and has been widely applied to behavioral decisions such as green consumption, environmental protection, and land transfer for farmers. However, given the complexity of the subject's behavioral influence, numerous empirical results show that the three main factors in TPB have a predictive power of 30%–40% for BI, and a relatively limited explanatory power for individual behavior. Therefore, Ajzen argues that TPB itself is an open model for behavioral research and that the original model can be extended and improved if other variables can significantly predict individual behavior [9]. The TPB model has been used in conjunction with the technology acceptance model (TAM) to study individual intentions and behaviors toward the acceptance and use of information technology [10–12]. More studies have extended factors involving cognition to TPB for broader research on of behavioral intentions, such as ecological environment perception, perceived risk, and trust [13–15].

The article "Function Mechanism of Psychological Driving Factors and Professional Transformation: Migrant Workers to Industrial Workers" was published in 2022. Journal: J Environ Public Health.

The study of risk perception first began in the 1960s and originated from people's irrational perception of risky behavior. Slovic, a foreign scholar, believes that risk perception is an individual's intuitive judgment of a risky event, an assumption about its possible outcome and impact, such that appropriate defensive measures can be taken in advance [16]. On the basis of Slovic's definition of risk perception, Chinese scholars put forward that risk perception refers to an individual's subjective feelings and understanding of various objective risks in the environment. Academia generally agrees on a strong link between risk perception and behavior. Initially, research on risk perception mainly focuses on safety behavior [17], of which worker safety is the main research object. In the British study on the risk-taking behavior of dump truck drivers on construction sites, risk perception has a significant impact on risk-taking behavior [18]. On miners' safety behavior, risk perception and self-control form a double mediator [19]. Risk perception is also applied to traffic, medical, and other safety behaviors. With the expansion of its scenarios, the application of risk perception in academia is not only limited to the prevention of dangerous behaviors but also applied to decision making of economic behaviors. On issues such as the choice of pension, and in organizational behavior management, managers' risk perception has a significant effect on organizational performance and enterprise innovation [20, 21]. Perception has a chain effect on the deposit trust mechanism of individuals [22], and those of pension risks are multidimensional and varied [23].

The essence of the professionalization behavior of migrant workers in the construction industry is the transformation and decision making of their own professional identity. The behavior itself is controlled by personal will. Risk perception is the individual's attitude and intuitive judgment on social risks. In the labor market, migrant workers themselves are more risk-aware. For high groups, risk perception also has a certain influence on behavioral decision making. Existing empirical studies have integrated risk perception into TPB theory. Zhang et al. analyzed the role of risk perception in influencing the consumer intentions of recycling mobile phones based on TPB theory [24]. Mullan et al. added risk perception to TPB theory to measure the safe handling of food by adolescents in the United Kingdom and Australia [25]. On this basis, this study incorporates the moderating factor of risk perception based on TPB and explores the psychological driving mechanism of professionalization of migrant workers in the construction industry, providing empirical evidence to explain and predict their decision making of professionalization behavior, and follows the principle of internal and external synergy to promote such professionalization.

The article "Function Mechanism of Psychological Driving Factors and Professional Transformation: Migrant Workers to Industrial Workers" was published in 2022. Journal: J Environ Public Health.

## 3. Research Hypothesis

As a mature theory in sociology, TPB is widely used to predict individual behavior. Numerous empirical studies have proven that this model can well explain the complexity of “will-behavior” of individuals, which is consistent with the logic of behavioral decision making of migrant workers in the construction industry.

### 3.1. Effect of Behavioral Attitude on Behavioral Intention

The professional attitude of migrant workers in the construction industry refers to their positive or negative attitude toward professional behavior. On the one hand, behavioral attitude is affected by one's own emotional attitude and is affected by instrumental and emotional attitudes, that is to say, whether this behavior is beneficial and can cause happiness. TPB points out that an individual's behavioral attitude has a significant positive effect on BI; that is, the more positive and supportive an individual attitude, the easier it is to produce a certain BI. By contrast, when an individual attitude is more disgusting and negative, the tendency to form actual behavior is also weaker. The increase in income after professionalization can significantly improve the enthusiasm of migrant workers for such transformation [26], and high salary also affects their intention to move [27]. In terms of the benefits and value brought about by behavior, the more positive the attitude toward it, the stronger the intention to act. Thus, the following hypothesis is proposed:

  Hypothesis 1: the professional behavior attitude of migrant workers in the construction industry has a positive impact on their BI.

### 3.2. Effect of Subjective Norm on Behavior Intention

Subjective norm refers to the social pressure that an individual feels about taking a certain behavior, that is, for the professionalization of migrant workers, the degree of influence of groups or individuals that affect the behavior of migrant workers on professionalization. TPB states a positive correlation between AT and BI. A more important subjective norm represents a stronger social influence, resulting in a higher tendency to implement the behavior. The level of family support and the surrounding relatives and friends engaged in the construction industry affect the professionalization of migrant workers [28]. The family and friends' encouragement and AT affect individual cognition [29], which can promote the enthusiasm for professionalization intention. Thus, the following hypothesis is proposed:

  Hypothesis 2: the subjective norm of the professionalization of migrant workers in the construction industry has a positive impact on their BI.

The article "Function Mechanism of Psychological Driving Factors and Professional Transformation: Migrant Workers to Industrial Workers" was published in 2022. Journal: J Environ Public Health.

### 3.3. Effect of Perceived Behavioral Control on Behavior Intention and Actual Behavior

PBC reflects the individual's controllability of implementing behaviors based on past experience and their own abilities. Ajzen believes that PBC may change with the situation. Each individual has its own education and living environment, and the factor of perceived behavioral control also profoundly reflects individual differences. PBC refers to the degree to which migrant workers feel control when they adopt professional behaviors, including internal factors (such as personal shortcomings, skills, abilities, or emotions) and external control factors (such as information and opportunities), and dependence or obstacles to others. In the literature, the judgment of a new generation of migrant workers on whether they can successfully complete a certain task significantly and positively affects their acquisition of professional ability [30]. Therefore, the more resources and opportunities of migrant workers in the construction industry believe they have at their disposal, the fewer obstacles to expect, and the stronger the intention to professionalize. Similarly, a survey of migrant workers found that their self-conditions, such as educational, professional, and technical levels, are highly important. Professionalization intention produces positive effects. The more capable you are and the more important you are to your career development, the stronger your intention to professionalize will be [31]. On this basis, the perceived behavioral control of migrant workers in the construction industry affects their professionalization intention and can also directly affect their professionalization behavior. Thus, the following hypotheses are proposed:

  Hypothesis 3: perceived behavioral control has a mediating effect on the professionalization intention of migrant workers in the construction industry.
  Hypothesis 3a: perceived behavioral control has a positive effect on the professionalization intention of migrant workers in the construction industry.
  Hypothesis 3b: perceived behavioral control has a positive effect on the professionalization behavior of migrant workers in the construction industry.

The article "Function Mechanism of Psychological Driving Factors and Professional Transformation: Migrant Workers to Industrial Workers" was published in 2022. Journal: J Environ Public Health.

### 3.4. Effect of Behavior Intention on Behavior

BI refers to the tendency of migrant workers in the construction industry to have professional behaviors. Numerous empirical studies have shown that individual intention is an important factor affecting behavior. Cristeam and Gheorghiu believed that BI is the premise of immediate action [32]. Fu et al. argued that individuals' stereotypical negative perceptions can produce irrational rejection behavior [33]. For promoting the professionalization of the construction industry, individual will is an important basis and also plays an important role in predicting the professionalization behavior. The intention of migrant workers has always been regarded as an important part of related research, and the positive impact of their training intention on behavioral enthusiasm has been confirmed [34]. The intention of migrant workers to become professionals directly affects their related behavior. Although the behavior is also affected by several external factors, combining these with control factors and the internal behavior intention can lead to actual professional behavior. Thus, this study proposes the following hypothesis:

  Hypothesis 4: the professionalization intention of migrant workers in the construction industry has a positive impact on their professionalization behavior.

### 3.5. Moderating Effect of Risk Perception

Numerous empirical results show that the three main factors in TPB have only 30%–40% predictive power for BI, and even more limited explanatory power for individual behavior. Therefore, TPB still needs to be supplemented and explored. Risk perception is an individual's attitude and subjective judgment about the effect of external objective risks on oneself. The decision making of the professionalization of migrant workers is actually under the context of risk conditions, which is more prominent in the construction industry. The project system of the construction industry is the source of the instability of migrant workers' occupation, and many of its risk factors affect farmers. When choosing a career development, migrant workers actually have characteristics of “rational people” [35]; that is, they compare and judge their own abilities, future risks and benefits, and take corresponding measures. However, migrant workers are affected by factors such as their own cultural quality, and their decision making cannot be completely rational. In addition, cognitive biases such as conformity and representative inspiration may occur. Therefore, the perception of risk affects their behavior. The majority of migrant workers are risk averse, and the more they perceive risks, the less likely their behaviors occur. Thus, this study proposes the following hypothesis:

  Hypothesis 5: risk perception can effectively moderate the influence of professional BI on behavior.

The article "Function Mechanism of Psychological Driving Factors and Professional Transformation: Migrant Workers to Industrial Workers" was published in 2022. Journal: J Environ Public Health.

To more visually demonstrate the hypothesized relationships among the factors, Figure 2 shows the model framework for the above proposed hypotheses.

## 4. Research Method

### 4.1. Measures and Questionnaire Design

Based on the above theoretical analysis, 21 indicators were designed in this study to measure six latent variables such as behavioral AT, SN, PBC control, BI, risk perception, and professionalized behavior (see Table 1) [38]. The behavioral AT scale was designed with reference to Chan's maturation scale. Starting from two dimensions of affective and instrumental attitudes, combined with relevant research on construction workers by scholars such as Yang and Chen [31, 36, 37], instrumental attitudes respond in terms of the growth of material economy and the degree of integration of life into the city. SNs are measured around support from family, leaders, workers, and the government [28, 29]. Perceived behavioral norms are developed from both self-efficacy and control perspectives, with reference to the scales of Carmeli, Schaubroeck, and Taylor and Todd [39, 40]. The measurement of risk perception, based on Slovic's research, is centered on the fearfulness of risk, that is, on possible behavior or decision consequences [16]. Measures of professionalization intention and behavior are mainly based on Chinese research on the professionalization of migrant workers in the construction industry [41, 42].

To ensure quality, we designed the questionnaire in accordance with the 10 principles such as clarity, singularity, and neutrality proposed by Zhong and Huang [43]. A small-scale professional prestudy was carried out before starting the large-scale formal questionnaire research, using a 5-point Likert scale to evaluate the actual situations according to the questions. The purpose of the 5-point scale was to allow migrant workers to easily understand the questions and to obtain more accurate data. The initial questionnaire consisted of 21 questions and took approximately eight minutes to complete, which falls within the acceptable range of the research participants. All 120 questionnaires were returned to the researcher, site manager, and university research faculty. Among the questionnaires, 12 with missing information and 4 with duplicate answers were excluded, yielding 104 valid questionnaires. Churchill believed that to test whether the structure of a questionnaire meets the requirements [44], the CITC needs to be tested. The common threshold value is 0.4 in academia, and after the reliability and CITC value tests, all the initial items are retained. The questionnaire content expression and item layout are further modified to form the official questionnaire, as shown in Table 1.

The article "Function Mechanism of Psychological Driving Factors and Professional Transformation: Migrant Workers to Industrial Workers" was published in 2022. Journal: J Environ Public Health.

### 4.2. Sample Selection and Data Sources

The questionnaires were mainly distributed through on-site surveys. Three cities with relatively high levels of economic development within China were selected based on GDP data: Nanjing, Jiangsu Province; Nantong, Jiangsu Province; and Hefei, Anhui Province. The reason why Jiangsu Province ranked first in the country in terms of economic GDP in the construction industry in 2021 was Nantong and Nanjing being the top two cities in this industry, representing its advanced development in China. In 2021, the year-on-year growth rate of construction GDP in Anhui Province is the second in China. With half of the construction GDP coming from Anhui Province, Hefei has a strong driving force for the development of this industry. The above survey target cities all have a high-level construction industry development. In terms of the professional development of construction workers, Anhui is one of leaders in the country. The survey samples can more fully reflect the will of the questionnaire. From the 422 questionnaires distributed on the spot, 19 with incomplete options, 11 with multiple choices, and 9 with answers that clearly did not meet the meaning of the question were deleted. Thus, 383 valid questionnaires were recovered, with an effective rate of 90.8%, which met the requirements for sample size and characteristics. The data characteristics of the sample are shown in Table 2.

## 5. Data Analysis and Results

### 5.1. Scale Reliability and Validity Test

As the data in Table 3, it shows that migrant workers in the construction industry hold relatively positive AT, SN, PBC, RP, BI, and B toward professionalism as a whole, with large variability among individuals. The reliability test uses the Cronbach's alpha coefficient calculated by SPSS22.0 as a measurement index. The resulting Cronbach's alpha coefficient of all latent variables is greater than 0.7 [45], indicating good reliability.

The results of validity analysis showed that the value of KMO was 0.826, and the cumulative variance contribution rate was 66.736% through Bartlett's test of sphericity (in Table 4), indicating that the index was suitable for factor analysis and had good reliability.

The article "Function Mechanism of Psychological Driving Factors and Professional Transformation: Migrant Workers to Industrial Workers" was published in 2022. Journal: J Environ Public Health.

Confirmatory factor analysis (CFA) showed that the standard loading coefficients of all indicators were significant. The values of the average variance extracted (AVE) corresponding to the six factors were all greater than 0.5 [46], and the composite reliability (CR) index was all higher than 0.7 [47], indicating high convergence (in Table 5).

### 5.2. Model Fit Test

To determine the fit validity of the overall model and the parameter estimates [48], we refer to Wu Minglong's evaluation, absolute fitness, value-added fitness, and the parsimonious fitness indexes.  Table 6 shows the test results. After inspection, all indicators meet the requirements, and the model fitting degree is good, indicating no further correction is required.

### 5.3. Model Test Results

#### 5.3.1. Direct Path Analysis

The direct hypotheses were examined by path analysis with structural equation models.  Table 7 and Figure 3 show the estimation results. AT, SN, and PBC have a significant positive effect on BI, with PBC having the largest path of effect. Thus, hypotheses 1, 2m, and 3a are supported. PBC and BI have significant positive relationship with B, and thus, hypotheses 3b and 4 are also supported. The results of the direct path illustrate the good adaptability of TPB in the study of the professionalization behavior of migrant workers in the construction industry.

#### 5.3.2. Mediation Effect Analysis

On the basis of the direct effect, this study further explores the mediating effect of PBC on B through the role of BI. To increase the accuracy of research results, this study uses bootstrap method to test the mediating effect.  Table 8 shows the results, and the confidence intervals of the total, direct, and indirect effects of PBC on B are satisfied. Thus, BI is a mediating variable of PBC on B and produces a partial mediating effect. Hypothesis 3 is proven valid.

#### 5.3.3. Analysis of Moderating Effects

In testing the moderating effect of risk perception, we refer to Zhonglin Wen and Yan Wu et al. [49], where the measurement terms were combined to form and assign values to the interaction terms based on the results of the CFA one-way test. Eventually, new estimation paths were defined for the model in AMOS, followed by corrections to the standardized coefficients of the interaction terms. To ensure the fit of the new model, recalculations were carried out and corrected according to the results using the MI error correction model. A path was created between residuals 5 and 6 to improve the NFI of the original model. The results of the moderating effects of the modified model are shown in Table 9.

The article "Function Mechanism of Psychological Driving Factors and Professional Transformation: Migrant Workers to Industrial Workers" was published in 2022. Journal: J Environ Public Health.

The data show that the interaction item (RP*∗*BI) has a significant moderating effect on the B of migrant workers in the construction industry. The standardization coefficient is −0.225, and the paths were all less than 0.01 with a high level of significance; that is to say, when the risk perception level of migrant workers is strong, the positive influence of behavior intention on behavior declines. RP acts as a negative moderator of the action relationship between BI and B. Therefore, Hypothesis 5 is supported.

### 5.4. Analysis of Results

The above empirical study of the professionalization behavior of migrant workers in the construction industry reflects the relationships and pathways of action between AT, SN, PBC, risk perception, and BI and behavior, with the Hypothesis 2 following specific findings.

1. The professional AT of construction migrant workers has a significant positive effect on BI, with the standardized path coefficient of 0.133. Compared with other factors, AT does not play a strong role in determining professional BI. The empirical evidence shows that BI depends on instrumental and affective attitudes. In addition, in career transition, migrant construction workers pay more attention to instrumental attitudes, especially the economic value that professionalization can bring, and their factor loadings are the largest.
2. SN has a significant positive influence on behavioral intentions, confirming with a standardized path coefficient of 0.138. The SN of migrant workers in the construction industry is mainly influenced by factors such as family members, surrounding workers, leaders, and the government. Among these, family members and the government play an important role in the formation of SN with a loading coefficient of 0.76.
3. PBC of migrant workers in the construction industry has the strongest positive effect on BI and has a significant positive effect on behavior. After empirical testing, PBC has a partial mediating effect on behavior through BI, but the indirect effect accounts for a low proportion of the total effect. Therefore, the direct path effect of PBC on BI is more important, confirming hypotheses 3, 3a, and 3b. PBC is mainly expressed in two aspects, namely, behavioral control and self-efficacy. The empirical results show that behavioral control, that is, the ability of migrant workers to solve problems in the career transition, has the strongest effect on PBC, with a loading coefficient of 0.79.
4. BI has a significant positive effect on B, confirming Hypothesis 4, which also verifies the role of psychological perceptions in driving behavior on professional transition. In the decision making of professionalization behavior in the construction industry, the stronger the BI of migrant workers, the more likely that professionalization behavior occurs. For the intention to professionalize behavior, compared with factors such as stable labor relations and participation in training, migrant workers' intention to learn skills and norms plays an important influential role.
5. RP has a significant moderating effect on professionalization intention and behavior, confirming Hypothesis 5. According to the survey data, the RP of migrant workers for professionalization is at a medium level, and the empirical study confirms that the relationship between risk perceptions on BI and B has a negative weakening effect. In terms of professional behavior drive, the influence of psychological cognition on behavior decreases at this time for migrant worker groups with high-risk perceptions. By contrast, the effect of psychological perception on behavior is increased for the low-risk perception group of migrant workers.

The article "Function Mechanism of Psychological Driving Factors and Professional Transformation: Migrant Workers to Industrial Workers" was published in 2022. Journal: J Environ Public Health.

## 6. Discussion

Given that relatively few psychological research mechanisms are available on the professionalization transition of migrant workers in the construction industry, this study aims to explore the key influencing factors and paths in their decision making. On the basis of expanding TPB, this study constructs a structural equation model and obtains a conclusion consistent with the previous hypothesis through empirical analysis. The professionalization behavior of migrant workers in the construction industry can be predicted by RP and BI. The empirical results show that AT, SN, and PBC play effective roles in predicting the formation of BI.

The present results find that in the actual work of the construction industry, PBC is an important factor affecting their intention to professionalize, which can indicate the importance of nonvolitional factors. The possible reason is that, on the one hand, migrant workers do not have the resources and opportunities (such as knowledge, ability, skills, and sufficient time) required for professionalization due to the limitation of educational background and professional skills. On the other hand, the career choice of farmers to become workers is significantly driven by profit, which perfectly matches their motivation to earn money to support their families. Thus, this motivation explains the important role of the family in predicting the intention to professionalize. Emotional attitudes such as love and enjoyment for construction work are therefore almost nonexistent, which also applies equally to the less controlled group. Therefore, the intention to professionalize of migrant workers can be effectively increased through education, training, and investment in resources and equipment.

The article "Function Mechanism of Psychological Driving Factors and Professional Transformation: Migrant Workers to Industrial Workers" was published in 2022. Journal: J Environ Public Health.

Several disadvantages in human capital investment of the construction industry migrant workers cause their weak ability to resist risks, and risk perception has a certain moderating effect when making behavioral decisions. Generally speaking, migrant workers are risk-averse and are more sensitive to the risk of economic loss driven by the purpose of working. Notably, migrant workers in the construction industry also attach great importance to the risk of legal constraints; they want to have more legal protection and at the same time want to bear as few legal obligations as possible. This psychological state of inequality of rights and obligations also stems from the confusion of the psychological contract between the enterprise and the migrant worker brought about by the customary governance of the construction industry. Therefore, the government, as a security agency, plays an important supporting role in managing the construction market and protecting the reasonable rights and interests of migrant workers. Therefore, the government must (1) regulate the labor market and balance the disadvantaged position of migrant workers in the employment market; (2) reconstruct the concept of labor contracts in the construction industry and strengthen the management of nonstandard employment; and (3) improve the social security system and clarify its own dominant position, adhering to the socialized operation of social security.

## 7. Conclusion

Construction migrant workers' career transition decision is a complex psychological cognitive process, and clarifying the psychological driving mechanism is important to effectively guide their professionalization behavior. Although TPB has been applied to behaviors such as green consumption and economic decision making, relatively limited research has been carried out on occupational behavior, and even less has been applied in relation to migrant workers. Based on this theory, this study fully combines the characteristics of construction industry and migrant workers, and innovatively introduces risk perception as a moderating variable to explore the cognitive driving mechanism that affects their professionalization behavior. From a large number of visits and research to obtain data, this study verifies the paths of AT, SN, PBC, and RP on the BI and B of migrant workers in the construction industry, empirically proving the theoretical applicability of professional behavior, and provides a guide for their professionalization transformation. Meanwhile, the findings further enrich the research on the vocational identity transformation of migrant workers in the construction industry. In terms of practice, identifying the psychological drivers of the professionalization behavior of migrant workers in the construction industry presents a guiding and facilitating role for the government to formulate policies and enterprises to improve management.

The article "Function Mechanism of Psychological Driving Factors and Professional Transformation: Migrant Workers to Industrial Workers" was published in 2022. Journal: J Environ Public Health.

This study adopts a more scientific and standardized empirical method, but retains several limitations. The questionnaire is based on scientific theories and beliefs, but many other factors affecting intention and behavior may be missing in the measurement of question items. Future research can extend the exploration to include more dimensional measures of the psychological mechanism of the professionalization behavior of migrant workers in the construction industry.

## Figures and Tables

**Figure 1:** Model diagram of TPB.

**Figure 2:** Conceptual model of research hypothesis.

**Figure 3:** Structural equation path diagram.

**Table 1:** Measures of factors influencing the professionalization of migrant workers in the construction industry.

Factor	Title number	Question item	References
Attitude	AT1	Professionalization can benefit me financially	Xiuli Yang & Lutang Li [31];
	AT2	Professionalization can facilitate urban integration	Min Chen [36];
	AT3	Professionalization is valuable	Ziyou Shen & Hong Feng [37];
	AT4	Professionalization is delightful	Chan [38]

Subjective norm	SN1	Families support their participation in professional transition	Jiayu Liu [28]; Limin Lv [29]
	SN2	Leaders believe that promoting professionalization must be carried out	
	SN3	The workers around me think that the professionalization must be promoted	
	SN4	The government issued a document to promote professionalization	

Perceived behavioral control	PBC1	I think I can successfully solve the obstacles to professionalization	Carmeli & Schaubroeck [39]; Taylor & Todd [40]
	PBC2	I think I have the knowledge and ability to professionalize	
	PBC3	I think I have the resources to professionalize (time, equipment, etc.)	

Risk reception	RP1	I am well aware that a fixed job position after professionalization may reduce income	Slovic [16]
	RP2	I am well aware that participating in professional training may take up labor time	
	RP3	I fully understand that participation in professionalization may be subject to legal constraints	

Behavioral intention	BI1	I am willing to learn career-related skills and norms	Xiuli Yang [41]; Zhanyuan Hou [42]
	BI2	I am willing to sign a labor employment contract with the company	
	BI3	I would like to participate in professional training on a regular basis	

Behavior	B1	Take work seriously and pursue work quality	Jiayu Liu [28]; Ajzen [7]
	B2	Always maintain a “safety first” work awareness	
	B3	Obtain the corresponding qualification certificate	
	B4	Perform work in accordance with operational specifications	

The article "Function Mechanism of Psychological Driving Factors and Professional Transformation: Migrant Workers to Industrial Workers" was published in 2022. Journal: J Environ Public Health.

**Table 2:** Statistical characteristics of the sample.

Characteristics	Sample size	Percentage (%)
Gender		
Male	284	74.2
Female	99	25.8

Age		
Under 30 years old	98	25.6
30–40 years old	124	32.4
40–50 years old	75	19.6
50–60 years old	68	17.8
60 years old and above	18	4.7

Educational background		
Primary school	89	23.2
Lower secondary	145	37.9
High school	88	23
University and above	61	15.9

Average annual income		
Less than 5 w	93	24.3
5–8 w	153	39.9
8–10 w	71	18.5
10–15 w	53	13.8
15 w or more	13	3.4

Number of school-age children		
0	33	8.7
1	102	26.6
2–3	146	38.1
3 or more	102	26.6

**Table 3:** Descriptive statistics and Cronbach's alpha.

Dimension	Variable	Descriptive statistics		Cronbach's alpha
		M	SD	
AT	AT1	3.77	1.099	0.819
	AT2	3.72	1.137	
	AT3	3.68	1.143	
	AT4	3.65	1.058	

SN	SN1	3.63	1.085	0.829
	SN2	3.65	1.121	
	SN3	3.73	1.14	
	SN4	3.69	1.118	

PBC	PBC1	3.71	1.08	0.765
	PBC2	3.73	1.13	
	PBC3	3.69	1.151	

RP	RP1	3.75	1.048	0.746
	RP2	3.78	1.118	
	RP3	3.68	1.176	

BI	BI1	3.77	1.143	0.747
	BI2	3.8	1.188	
	BI3	3.75	1.093	

B	B1	3.63	1.088	0.832
	B2	3.65	1.166	
	B3	3.75	1.163	
	B4	3.68	1.125	

**Table 4:** Results of Bartlett's test of sphericity.

Kaiser–Meyer–Olkin measure of sampling adequacy		0.826

Bartlett's test of sphericity	Approx. chi-square	4442.439
	df	210
	Sig.	0

**Table 5:** Results of convergent validity.

Dimension	Variable	Convergent validity		
		Standardized regression weights	CR	AVE
AT	AT1	0.808	0.822	0.538
	AT2	0.727		
	AT3	0.751		
	AT4	0.637		

SN	SN1	0.759	0.830	0.549
	SN2	0.724		
	SN3	0.723		
	SN4	0.758		

PBC	PBC1	0.787	0.766	0.523
	PBC2	0.696		
	PBC3	0.682		

RP	RP1	0.73	0.748	0.50
	RP2	0.656		
	RP3	0.73		

BI	BI1	0.826	0.755	0.510
	BI2	0.685		
	BI3	0.615		

B	B1	0.736	0.828	0.55
	B2	0.719		
	B3	0.786		
	B4	0.713		

*Note.* CR = composite reliability and AVE = average variation extraction.

**Table 6:** Model fit test.

Index	Absolute fit			Value-added fit index			Parsimonious fit index	
	*χ * ^2^/DF	RMSEA	GFI	NFI	CFI	IFI	PGFI	PNFI
Ideal value	<3	<0.05	>0.9	>0.9	>0.9	>0.9	>0.5	>0.5
Actual value	2.053	0.042	0.947	0.918	0.956	0.956	0.738	0.787

*Note. χ* ^2^/DF = Chi-square; RMSEA = root-mean-square error of approximation; GFI = goodness-of-fit index; NFI = normative fit index; CFI = comparative fit index; IFI = incremental fit index; PGFI=parsimony goodness-of-fit index; PNFI = parsimony-adjusted normed-fit index.

The article "Function Mechanism of Psychological Driving Factors and Professional Transformation: Migrant Workers to Industrial Workers" was published in 2022. Journal: J Environ Public Health.

**Table 7:** Direct path test results.

Hypothesis	Path	Estimate	S.E.	C.R.	*P*
H1	AT⟶BI	0.133	0.074	2.533	0.01
H2	SN⟶BI	0.135	0.058	2.604	0.009
H3a	PBC⟶BI	0.241	0.068	4.261	^*∗∗∗*^
H3b	PBC⟶B	0.206	0.055	3.781	^*∗∗∗*^
H4	BI⟶B	0.222	0.046	4.069	^*∗∗∗*^

*Note.* S.E. = standard error; C.R. = composite reliability. ^*∗∗∗*^Correlation is significant at 0.001 level.

**Table 8:** Mediation path test results.

Path	Point estimate	Multiplying coefficients		Bootstrapping			
		SE	Z	Bias-corrected 95% CI		Percentile 95% CI	
				Lower	Upper	Lower	Upper
Total effect							
PBC⟶B	0.261	0.061	4.279	0.151	0.391	0.261	0.387
Direct effect							
PBC⟶B	0.207	0.062	3.339	0.92	0.332	0.92	0.332
Indirect effect							
PBC⟶B	0.054	0.021	2.571	0.023	0.106	0.020	0.100

**Table 9:** Moderating effect test results.

Path	Estimate	S.E.	C.R.	*P*
RP⟶B	0.178	0.56	3.255	0.001^*∗∗*^
BI⟶B	0.181	0.45	3.288	0.001^*∗∗*^
RP^*∗*^BI⟶B	−0.225	0.50	−3.861	^*∗∗∗*^

*Note.* S.E. = standard error; CR = composite reliability. ^*∗∗*^Correlation is significant at 0.05 level. ^*∗∗∗*^Correlation is significant at 0.001 level.

## Data Availability

Data presented in this study are available from the corresponding author upon request.
